# Intelligent Community and Real Estate Management Based on Machine Learning

**DOI:** 10.1155/2022/7738811

**Published:** 2022-08-21

**Authors:** Zhixiao Ye, Yunlong Zhang, Juan Jiang, Tong Liu

**Affiliations:** ^1^School of Management, Zhejiang Shuren University and Institute of Modern Services, Hangzhou 310015, Zhejiang, China; ^2^Xi'an International University, Xi'an 710077, Shaanxi, China; ^3^Business School, Ludong University, Yantai 264025, Shandong, China; ^4^Property Management Department, School of Management, Zhejiang Shuren University, Hangzhou 310015, Zhejiang, China

## Abstract

When studying intelligent community and property management system, network service has an important impact on intelligent community construction and property management service. How to use machine learning and other technologies to improve the network service of intelligent community and integrate it into real estate property management is worthy of further research. This paper introduces the basic model of machine learning and proposes a network data prediction model based on time series. For the time dimension, an improved prediction algorithm model of machine learning is proposed. For mobile data allocation, from the perspective of ensuring the current and future continuity of the spectrum after spectrum allocation, this paper proposes a spectrum allocation algorithm based on the joint measurement of time domain and frequency domain. In addition, the VP-tree algorithm is used to construct the spatial vector relationship of the intelligent community. At the same time, in the time trend and periodicity of the mobile data in the intelligent community network, the attention mechanism is introduced to realize the distribution of mobile data and traffic prediction in the intelligent community by machine learning. This paper analyzes the requirements of the property management system, designs the property management information system including the field subsystem layer, data acquisition layer, and cloud service layer, introduces the property management module and customer service module in detail, and carries out the system test. The test results show that the system runs well. Finally, aiming at the problems existing in the property management industry, this paper puts forward the development strategy of property management.

## 1. Introduction

The rapid development of economy in the new era has led to the rise of intelligent communities. Intelligent communities use Internet of things and other technologies to meet people's convenience and intelligent needs for the living environment. For example, in aspects closely related to people, such as broadband mobile data and property management, they have become an important part of the development of intelligent communities [1, 2]. The distribution and setting of community mobile data directly affect people's sense of network use. At present, many researchers have carried out experimental research on the mobile data distribution technology of intelligent community [3]. Property management can reflect the service characteristics of urban communities and is also an important part of improving residents' well-being. Real estate property management can not only promote the real estate industry, but also further improve urban community services [4]. While continuously improving the service quality, it can expand from the field of life services to the field of culture and economy. With the continuous renewal of China's real estate economic system, in order to adapt to the market reform and the needs of consumers, real estate property management also presents diversified and industrialized development. However, the current property management enterprises have some problems, such as low service quality, nonstandard workflow, few service projects, and low professionalism of personnel. Therefore, the property management enterprises are small, unable to form large-scale development and poor enterprise benefits. The problems existing in real estate property management not only affect the rights and interests of consumers, but also hinder the development of real estate property management industry and intelligent community [5]. The improvement of consumers' awareness of rights protection and the reform of the real estate industry have gradually exposed the problems of the property management industry to the public. Therefore, the real estate property management industry is in urgent need of reform and development, and the development of intelligent community is also facing a new test [6, 7]. Based on the development needs of intelligent community, this paper studies the data distribution of community mobile network, puts forward the distribution data model and evaluation criteria, designs the intelligent community property management system, analyzes the problems existing in the current real estate property management industry, and puts forward the development strategy of intelligent community property management industry, so as to lay a theoretical foundation for the development of intelligent community and property management.

## 2. Related Work

The explosive growth of data and the improvement of computer technology have promoted the continuous development of intelligent community. Among them, the distribution of community network data and the prediction of traffic have become the focus of research. More and more researchers apply machine learning technology to mobile data distribution and traffic prediction. The literature proposes that the neural network prediction model has higher self-learning and adaptability compared with the traditional data statistics methods, and can adapt to the changing characteristics of large-scale data at any time [8]. Neural network is more practical in the field of traffic prediction, especially in the field of cyclic traffic prediction [9]. Therefore, more and more network traffic prediction methods use neural network. In the field of actual mobile network traffic, in addition to using the time dimension for research, it can also be predicted in the spatial dimension. According to the literature, according to the current characteristics of mobile network base station construction, if only the time characteristics are predicted, there are limitations [10]. Using the spatial sequence characteristics to predict the traffic can better meet the needs of mobile data base station design and planning. At the same time, it can further improve the intelligence of mobile data distribution. The literature proposes to predict and distribute community mobile network data based on machine learning method and spatio-temporal feature analysis [11]. The literature believes that although the time series and spatial series feature prediction models have been widely used, there are still some limitations [12]. It is more scientific to combine the two models to predict the traffic data. In terms of intelligent community property management, the literature believes that property management is an extended industry of real estate development and sales, and has gradually developed into a tertiary industry with independence and service. Property refers to the real estate industry. It is the management object of property management. The owner or consumer is the service object of property management. The service content includes management, operation, and business. Property management is a paid service activity. Literature holds that property management refers to the management and service of the living environment by consumers through authorization and entrustment and through the relevant management mode or technology adopted by a third-party professional organization or organization [13]. According to the literature, property management is to manage the safety, environmental greening, road maintenance, and sanitary cleaning around consumers, and provide certain services to owners or consumers according to the contents of the contract. It is a service for the whole life cycle of buildings, from the early stage to the middle stage, and from the design and maintenance of buildings to the whole life cycle of buildings. The literature puts forward that property management belongs to organized and regular business activities [14]. The operating company achieves the purpose of making profits by creating a service value, selling the value to customers, and maintaining the long-term service relationship between property companies and consumers. With the continuous development of market economy and information technology, the marketing means of property management has shifted from offline to online [15]. At the same time, providing network services is also a new direction of property management development. Network service is the integration of traditional property management and emerging information technology, and has become an important service content of property management in intelligent community.

## 3. Machine Learning Technology

### 3.1. Basic Model

Whether the prediction result of machine learning model is accurate is usually measured by evaluation index. RMSE can compare the predicted value with the actual value. The formula is

(1) $$\begin{array}{c} \text{RMSE}=\sqrt{\frac{1}{N}\sum_{t=1}^{N}{\left(x_{t}-y_{t}\right)}^{2}.} \end{array}$$

MAE can reflect the actual situation of predicted value error, and the formula is as follows:

(2) $$\begin{array}{c} \text{MAE}=\frac{1}{N}\sum_{t=1}^{N}\left|\left(x_{t}-y_{t}\right)\right|. \end{array}$$

ARIMA is a time series prediction model, which takes into account the random fluctuation of time series. The formula is as follows:

(3) $$\begin{array}{c} X_{t}=\alpha_{1}X_{t-1}+\alpha_{2}X_{t-2}+\alpha_{p}X_{t-p}+\varepsilon_{t}+\beta_{1}\varepsilon_{t-1}+\ldots +\beta_{q}\varepsilon_{t-q}. \end{array}$$

The classical time series decomposition method based on moving average is realized by using additive model or multiplicative model on the premise that the periodic factors of time series are roughly consistent in each decomposition cycle. Among them, the concept of m-order moving average is used, that is,

(4) $$\begin{array}{c} {\hat{T}}_{t}=\frac{1}{m}\sum_{j=-k}^{k}y_{t}+j. \end{array}$$

Sequence decomposition algorithm based on additive model: assuming that the time series is *y* (t), the additive model of the sequence is expressed as follows:

(5) $$\begin{array}{c} y\left(t\right)=S\left(t\right)+T\left(t\right)+r\left(t\right). \end{array}$$

*S*(*t*) represents the periodic component of the sequence, *t*(*t*) represents the trend term of the sequence, *R*(*t*) represents the residual part after sequence decomposition, and the remaining residual is

(6) $$\begin{array}{c} r\left(t\right)=y\left(t\right)-T\left(t\right)-S\left(t\right). \end{array}$$

Sequence decomposition algorithm based on multiplicative model: assuming that the sequence is *y*(*t*), the additive model is as follows:

(7) $$\begin{array}{c} y\left(t\right)=S\left(t\right)+T\left(t\right)+r\left(t\right). \end{array}$$

*S*(*t*) represents the periodic component of the time series, *T*(*t*) represents the trend term of the time series, *R* (*t*) represents the residual part of the time series after decomposition, and the remaining residual is

(8) $$\begin{array}{c} r\left(t\right)=y\left(t\right)-T\left(t\right)-S\left(t\right). \end{array}$$

For the decomposed time series, the trend and periodicity of the original time series can be analyzed by adopting specific formulas. The time series decomposition algorithm of additive model has the following definitions:

(9) $$\begin{array}{c} F_{T}=\max\left(0,1-\frac{\text{Var}\left(R_{t}\right)}{\text{Var}\left(T_{t}+R_{t}\right)}\right),\\ F_{S}=\max\left(0,1-\frac{\text{Var}\left(R_{t}\right)}{\text{Var}\left(S_{t}+R_{t}\right)}\right). \end{array}$$

### 3.2. Community Mobile Data Distribution Algorithm

For the mobile network data allocation of the intelligent community, the location where the service can be allocated can be found through the candidate spectrum block, and then the time-domain fragment generated by the current service allocation can be calculated according to the remaining duration of adjacent services. The time fragment measurement formula is as follows:

(10) $$\begin{array}{c} \text{TFM}\left({\text{Link}}_{{\text{CSB}}_{i,j}}\right)=\left\{\begin{array}{c} 1\;t_{0}\leq \tau_{\text{adj}}\\ 1+\Delta \tau /t_{0}t_{0}>\tau_{\text{adj}} \end{array}.\right) \end{array}$$

The above formula is used to evaluate the impact of allocating services at the link on the original link in the future frequency domain. If the service is divided in a position that just meets the required number of frequency slots, the service has two adjacent services. At this time, only the TFM with the adjacent service with the longest remaining duration is calculated. The specific situation of TFM can be shown in Figure 1.

In order to explore the carrying capacity of the link, define the spectrum continuity of the link:

(11) $$\begin{array}{c} \text{LSC}\left(\text{Link}\right)=\frac{\sqrt{\sum_{i\in \text{Link}}{\left|{\text{Block}}_{i}\right|}^{2}}}{N}. \end{array}$$

Spectrum continuity change measurement SCVM definition:

(12) $$\begin{array}{c} \text{SCVM}\left({\text{Link}}_{{\text{CSB}}_{i,j}}\right)=\frac{{\text{LSC}}_{\text{bef}}\left(\text{Link}\right)-\text{LSC}\left({\text{Link}}_{{\text{CSB}}_{i,j}}\right)}{{\text{LSC}}_{\text{bef}}\left(\text{Link}\right)}. \end{array}$$

This paper introduces a time-frequency domain joint measurement index of link:

(13) $$\begin{array}{c} \text{TSCM}\left({\text{Link}}_{{\text{CSB}}_{i,j}}\right)=\text{TFM}\left({\text{Link}}_{{\text{CSB}}_{i,j}}\right)*\text{SCVM}\left({\text{Link}}_{{\text{CSB}}_{i,j}}\right). \end{array}$$

Under the condition that the existing spectrum resource occupation information remains unchanged, the service allocation at the end of the link will affect the future carrying capacity of the link to a certain extent, which is specifically reflected in the formation of new spectrum fragments in the future due to the difference of duration, which will affect the future continuity of the link. Therefore, the service should be allocated where the duration is less than that of adjacent services as far as possible, and the continuity of the original link should be affected as little as possible. Therefore, the smaller the TSCM value, the smaller the impact of service allocation on the current link, and the more reasonable the allocation scheme. Generally, spectrum allocation is performed on path *P* containing multiple links, so the time-frequency domain joint measurement index of path *P* is

(14) $$\begin{array}{c} \text{TSCM}\left(P\right)=\frac{\sum_{\text{Link}\in P}\text{TSCM}\left(\text{Link}\right)}{\left|L_{P}\right|}. \end{array}$$

### 3.3. Prediction Analysis and Simulation

The method proposed in this paper constructs the spatial combination by looking for the adjacent cells within m meters of the target cell. VP-tree is a binary tree structure that measures the space based on the distance information. It mainly uses the distance information between the commanding point and the target point to divide the space. For the calculation of the distance between cells, the longitude and latitude information of the cell can be used. Since the Earth is a spherical surface, the calculation of longitude and latitude should also be considered on a spherical surface, which can be calculated by haversine formula:

(15) $$\begin{array}{c} \text{haver}\sin\left(\frac{d}{R}\right)=\text{haver}\sin\left(\varphi_{2}-\varphi_{1}\right)+\cos\;\varphi_{1}\cos\;\varphi_{2}\text{haver}\sin\left(\lambda_{2}-\lambda_{1}\right),\\ \text{haver}\sin\left(\theta \right)=\sin^{2}\left(\frac{\theta }{2}\right)=\frac{\left(1-\cos\left(\theta \right)\right)}{2}. \end{array}$$

After forming a cell spatial binary tree by constructing VP-tree, you can quickly find several cells within a specified distance next to any target cell. In fact, the attention mechanism is to add an attention layer after the encoder to calculate the similarity between each expected input of the encoder and each time point of the encoder, to obtain an attention matrix. In the decoding process of the encoder, the predicted output of each time point corresponds to different context variables, so it will reflect a better trend, as shown in Figure 2.

The processing of each vector at the encoder and decoder layer is as follows:

Encoder:

(16) $$\begin{array}{c} h_{i}=\tanh\left(W\left[h_{i-1},x_{i}\right]\right),\\ o_{i}=\text{soft}\max\left(Vh_{i}\right). \end{array}$$

Decoder:

(17) $$\begin{array}{c} C_{t^{\prime }}=\sum_{i=1}^{T}\alpha_{t^{\prime }i}h_{i},\\ \alpha_{t^{\prime }i}=\frac{\exp\left(e_{t^{\prime }i}\right)}{\sum_{i=1}^{T}\exp\left(e_{t^{\prime }{}_{k}}\right)},\\ e_{t^{\prime }i}=v_{d}^{T}\tan\;h\left(W_{d}\left[d_{t^{\prime }-1};h_{i}\right]\right). \end{array}$$

The traffic prediction of intelligent community will produce different information sequences due to its own time and space factors, which are closely related, and working days, rest days, or weather factors may affect the prediction of mobile data traffic sequences. Therefore, by comprehensively considering external factors and based on embedding coding technology, this paper constructs a mathematical model integrated with neural network:

(18) $$\begin{array}{c} \text{Embedding}l_{g}=w_{g}\cdot l_{g}. \end{array}$$

The hidden state changes of each LSTM unit of the decoder are as follows:

(19) $$\begin{array}{c} d_{t^{\prime }}=f_{d}\left(d_{t^{\prime }-1},\left[{\hat{y}}_{t^{\prime }-1}^{i};ex_{t^{\prime }};c_{t^{\prime }}\right]\right). \end{array}$$

Predicted value:

(20) $$\begin{array}{c} {\hat{y}}_{t^{\prime }}^{i}=v_{d}^{T}\left(W_{m}\left[c_{t^{\prime }};d_{t^{\prime }}\right]+b_{m}\right)+b_{y}. \end{array}$$

The loss function in the training process adopts MSE as the error calculation formula, which is expressed by mathematical symbols and can be defined as

(21) $$\begin{array}{c} \text{loss}=\frac{1}{n}\sum_{i=1}^{n}{\left({\hat{y}}_{i}-y_{i}\right)}^{2}. \end{array}$$

A section of traffic data is randomly selected in the data test set for verification. The comparison between the predicted traffic value and the actual value of the algorithm proposed in this paper is shown in Figure 3.

## 4. Design of Intelligent Community Real Estate Property Management System

### 4.1. System Requirements Analysis

The system can improve the operation and management ability of the property management company, especially in commercial marketing, property management, and advertising investment. Only by improving the operation and management ability can we improve the overall competitiveness of the company. In addition, property companies also need to standardize human management, financial management, and other aspects, further improve personnel management and organizational planning ability, form the company's organizational advantages, and build the company's brand value.

The system can help enterprises expand their business scale. Only if they have high abilities in investment analysis and business expansion, and have the ability to analyze and learn market analysis and dynamic research, they can help managers improve the company's business planning ability and further expand the company's business scale.

The system has a high level of information technology operation and management. At present, computer technology, Internet of things, and other technologies are developing rapidly. In terms of intelligent community construction and property management, a variety of emerging information technologies need to be used to meet various needs of consumers, especially network services. At the same time, the system also needs to meet the remote communication of multiple offline management institutions, realize real-time communication, give play to the effect of face-to-face communication, and improve the company's cross-regional management ability.

### 4.2. System Structure Design

The structure of the intelligent community property management system proposed in this paper is shown in Figure 4. The system is divided into three layers: field subsystem layer, data acquisition layer, and cloud service layer.

The software architecture of the system is divided into five layers: data presentation layer, business logic layer, data cache middleware layer, data logic layer, and data adaptation layer. The specific architecture is shown in Figure 5.

### 4.3. System Function Design

#### 4.3.1. Property Management

The property management module is the most important functional module in the system designed in this paper, which can realize all kinds of property management and service work of the property company. This module can sort out and collect the information of houses, owners, environment, and equipment in the charge of the company. Through the function of this module, the property service can be realized, the problems between property companies, real estate companies, and residents can be handled, and the relationship between consumers and companies can be maintained. At the same time, it can help property management companies realize standardized property management and further improve consumers' sense of happiness and experience.

#### 4.3.2. Customer Service Management

The service cycle of customer service management is longer, the complexity is higher, and higher professionalism is required. Generally, high-quality customer service can only obtain certain economic benefits after a long period of time, so the company needs a more standardized information system to help the company complete the content of customer service management. Now more and more companies pay attention to customer service management. The customer service management function designed by this system can help enterprises comprehensively and timely grasp the effect of customer service management, and can make reasonable planning and timely adjust the content of customer service management. This module designs a reminder mechanism and collaborative office mechanism, which can help managers obtain real-time customer information, timely understand customers' needs or problems reflected in property management, reply and deal with consumers' questions or suggestions, and establish a feedback mechanism to further improve consumers' trust in property management companies.

### 4.4. Database Design

The system uses MySQL database to store user and business information, and the user information is shown in Table 1.

The specific information of user role is shown in Table 2.

Residential complaints and property reply forms are the problems of preserving residential complaint communities. The detailed design is shown in Table 3.

### 4.5. System Test

For the physical management system of intelligent community, the system is tested through information change, query, and maintenance. The specific test environment is shown in Table 4.

The test results of some functions of the system are shown in Table 5.

## 5. Research on Property Management Strategy of Intelligent Community

### 5.1. Problems in Property Management

#### 5.1.1. Overall Service Level and Personnel Quality of the Industry Are Low

People's living standards are getting higher and higher, and they need high-quality property services to meet people's growing cultural and living needs. However, at present, most property companies can only provide simple property services, which cannot meet people's demand for high-quality property services. The overall service level of the property management industry is low. Some property companies have not found their own positioning, but still believe that property managers are managers rather than service providers, and have no service awareness, nonstandard management, and poor service quality, and there are problems of arbitrary charges. In addition, the property industry belongs to the service industry. The salary income of employees is low, the working hours are high, and the rest time is short. Some posts even need 24-hour operation. Moreover, the society has a certain prejudice against the property service industry, resulting in the relatively low quality of employees in the industry, which is difficult to retain and attract high-level and high-quality talents.

#### 5.1.2. Mismatches between Property Management and Management of the Owners' Committee

At present, many communities or communities have not established owners' committees, or the owners' committees have formed interest alliances with property companies, resulting in that ordinary residents have no way to choose companies with better property services through democratic methods, resulting in nonstandard property management and inadequate property services. There are more and more contradictions and disputes between property companies and residents, and owners are unwilling to pay property fees, resulting in worse property service levels. Form a vicious circle.

#### 5.1.3. Difficult Administrative Supervision

At present, the administrative department for property management is understaffed and the administrative force is weak, but the supervision task is large, and there are some contradictions. Moreover, most administrative personnel are busy with daily affairs, the regulatory role is not obvious, and the administrative guidance is not in place. In the actual supervision work, the punishment of illegal enterprises is not high, and there is a problem of single management means. Some property companies infringe on the interests of residents, and the administrative departments do not take the initiative to punish the property companies, or there is no basis for relevant laws and regulations. Some of the contradictions between the property company and the owner are that the performance of the contract is not in place, and some are illegal buildings. However, the administrative department has not formed a joint force in property management and supervision, so it is unable to properly solve the contradictions between the property company and the owner.

#### 5.1.4. Unpaid Property Fees Affect the Service Management Level

Due to a variety of reasons, most communities are in arrears of property management fees. At present, the government departments have issued guidance standards and rules and regulations related to property services, but in practice, residents may be dissatisfied with the health work of the property company, parking lot management, advertising and investment promotion of public parts, and other problems, and take this as a reason or excuse not to pay the property management fee. There are some residential areas due to the historical problems left over by the developers, the unfinished infrastructure construction, or property right certificate handling of the residential area, and the inadequate supporting equipment will also become the reasons for the owners to owe the property management fee. The property company has no source of income. The owners' arrears of property fees will directly affect the service level and service quality of the property company, and even affect the normal life of residents in serious cases.

#### 5.1.5. Owner Has Weak Awareness of Public and Autonomous Management

As Party A of property management, the owner has the right to supervise the property management and the obligation to perform the contract. Many owners do not actively participate in the construction of the owners' committee, lack the awareness of active participation, and do not perform the contract signed with the property company, which is prone to disputes with the property company. In addition, some owners have bad behavior habits and their personal quality needs to be improved, such as taking out garbage at will, occupying public passages, parking at random, building in violation of regulations, and damaging house structures. The owner's personal behavior will directly affect the normal development of property services. The owner's civilization and compliance with public regulations will directly affect the service level of the property company.

### 5.2. Property Management Strategy Selection

#### 5.2.1. Improve the system and Establish Property Management Laws and Regulations

First, we should improve the property service bidding management system and use market rules to regulate and restrict the behavior of property companies. Clarify the content of the property service contract, specify the main responsibilities, rights, obligations, and liabilities for breach of contract of the enterprise and the owner, further refine the property service level, and clarify the work content, service standard, and charging standard for each level of property service.

Second, we should establish and improve the legal system of property management. Relevant government departments should establish the archives of property management companies, establish the service quality evaluation system of property management companies, regularly assess the property companies, file the service quality of property companies, carry out standardized management of property management companies, and take the owner's satisfaction as an important reference for the bidding of property management companies.

Third, we should establish and improve the property complaint mechanism, clarify the supervision contents, investigate and deal with the nonstandard behaviors of property companies in time, and effectively protect the rights and interests of households and consumers. Property management should clarify the charging scope and charging standard, and the property management company should regularly announce the use of property management fees, such as building repair, road maintenance, public facilities maintenance, security work, cleaning work, and greening maintenance.

Fourth, we should improve the punishment mechanism of property companies and implement blacklist management. For those with poor service quality of property companies and more complaints from owners, the property management contract can be terminated in accordance with the regulations, and the satisfaction evaluation results of residents can be directly linked to the property management expenses, so as to further restrict the behavior of property management companies. Government departments should strengthen the investigation and punishment of property companies with poor service quality and cancel the qualification of companies with nonstandard management.

#### 5.2.2. Strictly Manage and Guide the Healthy and Sustainable Development of Property Management Enterprises

On the one hand, the top-level design of policies can help accelerate the development of the property service industry and further standardize industry standards, laws, and regulations. Government agencies can take various measures to cultivate more professional property management talents. Colleges and universities can set up property management-related majors to further do a good job in talent training. The property company can establish a school enterprise cooperation mode with colleges and universities. According to the needs of enterprises, the school can train professional talents suitable for the market demand by providing high-quality teaching. Government departments can also play a public welfare management function, set up job skills training related to property management, improve the quality of property practitioners, and carry out property service skills training in a planned and purposeful way every year. Through this targeted job training, the overall service level and professional level of the industry can be improved. Government departments can also set up a property service communication platform to promote learning and exchange between property companies. Property companies in different regions have accumulated a lot of property service experience in the process of practice. Government departments can help companies establish communication bridges, realize experience sharing and resource sharing, and promote the healthy development of the property industry. At the same time, we should guide all companies to establish brand service awareness, pay attention to brand construction and company image, create professional company brands, and promote benign competition among companies.

On the other hand, property companies should develop in the direction of specialization. Property companies need to investigate and analyze the owners, further understand the needs of the owners, and be able to provide different property services for different regions, different people, and different geographical locations. At the same time, we should actively listen to the opinions and suggestions of the owners, further sort out the problems existing in our own management, constantly improve innovation, improve service quality, meet the needs of the owners, broaden market channels, and explore potential services.

#### 5.2.3. Change the Concept and Expand the Depth and Breadth of Property Management Services

At present, most property services stay in the basic aspects of water and electricity maintenance, sanitation, and safety guarantee. These works cannot reflect the depth and breadth of property management, and cannot meet the needs of owners for high-quality property services. Therefore, property companies need to change the traditional management concept and further tap the potential value of property services. The owner's demand for property services is multi-level and all-round. In addition to the basic water, electricity, heating, and parking security, there are more cultural needs. Therefore, the property company can further explore the breadth of property services and expand new projects and services on the basis of traditional service contents. Property management companies need to make progress, update management mode, innovate working methods, develop in the direction of modernization, further provide high-quality services, refine property services, and make enterprises bigger and stronger.

## 6. Conclusion

The construction of intelligent community is inseparable from real estate property management. People have more and more demand for property management services and higher standards. Based on machine learning technology, this paper explores the new direction of property management services in intelligent community, constructs the mathematical model of mobile data flow prediction in machine learning network, and puts forward the method of network mobile data distribution. According to the time characteristics of mobile data, attention mechanism is introduced. The network mobile data service of intelligent community is realized. This paper analyzes the requirements of the property management system and designs the property management information system, which mainly includes the field subsystem layer, data acquisition layer, and cloud service layer. At the same time, it analyzes the problems existing in the current property management service industry, such as the low quality of employees in the industry, the small intensity of administrative supervision, and the weak awareness of joint participation of owners. Finally, it puts forward the development strategy of the property service industry. The government departments need to improve the relevant systems, establish the property industry standards, guide the property companies to change their ideas, further expand the depth and breadth of property management services, and guide the healthy and sustainable development of the property management industry.

## Figures and Tables

**Figure 1:** Example of spectrum allocation considering time dimension.

**Figure 2:** Attention mechanism.

**Figure 3:** Comparison between predicted value and actual value of VP-tree + attention model.

**Figure 4:** Overall structure of property management information system.

**Figure 5:** Overall architecture of property management information system integration platform.

**Table 1:** User information.

Field	Name	Data type	Remark
Id	Primary key	Int (11)	Self-increase
User_name	Name	Varchar (50)	Users register themselves
Password	Key	Varchar (50)	Users register themselves
Nick_name	Nick name	Varchar (50)	Users register themselves
Role_id	Role	Int (11)	Users register themselves
Phone_num	Contact information	Varchar (50)	Users register themselves
E-mail	E-mail address	Varchar (50)	Users register themselves
Create_time	Registration time	Timestamp	Record when registering
Update_time	Update time	Timestamp	Record during operation
Delete_status	Status display	Varchar (1)	Effective or invalid state

**Table 2:** User roles.

Field	Name	Data type	Remark
Id	Primary key	Int (11)	Self-increase
Role_name	Character name	Varchar (20)	Users register themselves
Create_time	Registration time	Timestamp (0)	Record when registering
Update_time	Update time	Timestamp (0)	Record during operation
Delete_status	Status display	Varchar (1)	Effective or invalid state

**Table 3:** Resident complaints and property replies form.

Field	Name	Data type	Remark
Id	Primary key	Int (11)	Self-increase
Title	Topic	Varchar (225)	Users register themselves
Content	Content	Varchar (225)	Users register themselves
URL	Picture	Varchar (50)	Related pictures
Create_time	Registration time	Timestamp (10)	Record when registering
Reply	Reply	Varchar (225)	Users register themselves
Role_id	Role	Int (11)	Users register themselves
Reply_time	Response time	Timestamp (0)	Record during operation
Status	Status display	Tinyint (1)	Revisible or un-wintering status

**Table 4:** System test environment information.

Test environment	Windows server
Development tools	Eclipse
Server	Tomcat
Test content	Based on system requirements and architecture design, testing the operation rate and logical process of data
Test range	Intelligent community real estate property management system

**Table 5:** System test results.

No.	Operate	Content	Result
1	New service content	New service matters page, fill in the relevant information, click the saving button	Pass
2	Modify the service content	Click the saved service items, and then click the modification button. After modifying the service content on the service matters, click the saving button	Pass
3	Query service list	Select the query keywords, query the service information list, and arrange the search content searched in accordance with the order of time	Pass
4	Owner information maintenance	Select the designated owner's information for maintenance, click the modification button to update or modify the information, and click the save button after modification	Pass
5	Maintenance of work order information	Select the complaint work order, click the modification button, reply on the work order information page, and click the saving button after the input is completed	Pass

## Data Availability

The data used to support the findings of this study are available from the corresponding author upon request.
